RETRACTED

# Alleviation of Inflammation and Oxidative Stress in Pressure Overload-Induced Cardiac Remodeling and Heart Failure via IL-6/STAT3 Inhibition by Raloxifene

**DOI:** 10.1155/2021/6699054

**Published:** 2021-03-20

**Authors:** Shengqi Huo, Wei Shi, Haiyan Ma, Dan Yan, Pengcheng Luo, Junyi Guo, Chenglong Li, Jiayuh Lin, Cuntai Zhang, Sheng Li, Jiagao Lv, Li Lin

**Affiliations:** ^1^Division of Cardiology, Department of Internal Medicine, Tongji Hospital, Tongji Medical College, Huazhong University of Science and Technology, Wuhan, China; ^2^Division of Cardiology, Department of Internal Medicine, First People's Hospital of Shangqiu, Shangqiu, China; ^3^Department of Medicinal Chemistry, College of Pharmacy, University of Florida, Gainesville FL, USA; ^4^Department of Biochemistry and Molecular Biology, University of Maryland School of Medicine, Baltimore MD, USA; ^5^Department of Geriatrics, Tongji Hospital, Tongji Medical College, Huazhong University of Science and Technology, Wuhan, China

## Abstract

**Background:**

Inflammation and oxidative stress are involved in the initiation and progress of heart failure (HF). However, the role of the IL6/STAT3 pathway in the pressure overload-induced HF remains controversial.

**Methods and Results:**

Transverse aortic constriction (TAC) was used to induce pressure overload-HF in C57BL/6J mice. 18 mice were randomized into three groups (Sham, TAC, and TAC+raloxifene, *n* = 6, respectively). Echocardiographic and histological results showed that cardiac hypertrophy, fibrosis, and left ventricular dysfunction were manifested in mice after TAC treatment of eight weeks, with aggravation of macrophage infiltration and interleukin-6 (IL-6) and tumor necrosis factor-alpha (TNF-*α*) expression in the myocardium. TAC (four and eight weeks) elevated the phosphorylation of signal transducer and activator of transcription 3 (p-STAT3) and prohibitin2 (PHB2) protein expression. Importantly, IL-6/gp130/STAT3 inhibition by raloxifene alleviated TAC-induced myocardial inflammation, cardiac remodeling, and dysfunction. *In vitro*, we demonstrated cellular hypertrophy with STAT3 activation and oxidative stress exacerbation could be elicited by IL-6 (25 ng/mL, 48 h) in H9c2 myoblasts. Sustained IL-6 stimulation increased intracellular reactive oxygen species, repressed mitochondrial membrane potential (MMP), decreased intracellular content of ATP, and led to decreased SOD activity, an increase in iNOS protein expression, and increased protein expression of Pink1, Parkin, and Bnip3 involving in mitophagy, all of which were reversed by raloxifene.

**Conclusion:**

Inflammation and IL-6/STAT3 signaling were activated in TAC-induced HF in mice, while sustained IL-6 incubation elicited oxidative stress and mitophagy-related protein increase in H9c2 myoblasts, all of which were inhibited by raloxifene. These indicated IL-6/STAT3 signaling might be involved in the pathogenesis of myocardial hypertrophy and HF.

RETRACTED

## 1. Introduction

Heart failure (HF) is suffered by 26 million people, and the prevalence was approximately 1-2% worldwide as estimated [1]. Hemodynamic overload, caused by aortic coarctation or hypertension, is one of the momentous pathological irritations of HF [2]. HF patients are often associated with cardiac hypertrophy and reduced myocardial compliance. To some certain people, the current drug-based management is limited or in vain to their remission. Several lines of evidence showed that chronic inflammation plays an important role in adverse cardiac remodeling and the development of HF. In HF patients, the levels of proinflammatory circulatory factors were increased, such as IL-6, TNF-*α*, CRP, GDF15, and galectin-4 [3]. In patients with chronic persistent systematic inflammation, such as rheumatoid arthritis [4], inflammatory bowel disease [5], or obesity [6, 7], the risk of cardiovascular disease, including HF, was higher than that in general people. However, the causal relationship between HF and inflammation is still confused.

Although the chimeric monoclonal antibody to TNF-*α* showed no benefit to patients with moderate-to-severe chronic heart failure [8], other research declared IL-6 exerted an important role in HF and was strongly associated with adverse outcome in HF patients [9, 10]. Interleukin-6, as a typical proinflammatory cytokine, forms a complex with IL-6 receptor (IL-6R) and coreceptor glycoprotein 130 (gp130), which in turn initiates a cascade reaction including Janus kinase (JAK) activation, phosphorylation of STAT3 (p-STAT3), and subsequent dimer formation, nuclear translocation, and gene transcription [11]. However, conflicting consequences of IL-6 deletion in transverse aortic constriction (TAC) mice were reported [12, 13]. The left ventricular remodeling after TAC of IL-6-knockout mice was reduced in the research of Zhao et al. [13], whereas left ventricular hypertrophy and dysfunction by TAC showed no difference between wild-type and IL-6-knockout mice according to Lai et al. [12]. Hence, the role of IL-6 in cardiac hypertrophy and HF is not definite.

Raloxifene is approved by the FDA for the prevention and treatment of postmenopausal osteoporosis [14]. It has been discovered as a novel inhibitor of the IL-6/gp130 interface recently and inhibits the phosphorylation of STAT3 in cancer cells in our previous studies [15, 16]. The protective effect of raloxifene in cardiac remodeling and dysfunction induced by pressure overload is contradictory as previous studies reported [17, 18]; moreover, the potential molecular mechanism and anti-inflammation effect of raloxifene in the cardiovascular system are unclear likewise. In this paper, we provided more evidence about whether IL-6/gp130/STAT3 signaling was activated in TAC mice and the cardioprotective mechanism of raloxifene on pressure overload-induced cardiac hypertrophy and HF.

RETRACTED

## 2. Materials and Methods

All experiments have been approved by the institutional review board of Tongji Hospital, Tongji Medical College, Huazhong University of Science and Technology.

### 2.1. Transverse Aortic Constriction Mouse Model

Wild-type C57BL/6J mice (male, about 8 weeks and 25 g) purchased from the Jackson Laboratory were randomized into three groups: Sham, TAC, and TAC+raloxifene (raloxifene) groups (*n* = 6). Raloxifene hydrochloride (HY-13738A, MedChemExpress, U.S.) was dissolved with dimethyl sulfoxide (DMSO) firstly and then diluted with phosphate buffer saline (PBS) containing 20% (20 *μ*g HPBCD/100 *μ*L PBS, 0.2 mg/mL) hydroxypropyl B cyclodextrin (HPBCD). Raloxifene (15 mg/kg) was given daily by intragastric administration to the raloxifene group three days before TAC surgery and continued till mice were sacrificed, while the Sham and TAC groups are supplied by solvent without raloxifene. A practiced single operator performed all surgical procedures of TAC for the experiments as described previously [19]. A 27^1/2^ gauge blunt needle was applied to perform TAC surgery, and the Sham group was conducted with the surgery without tied tightly around the aortic arch against a cannula. After 4 or 8 weeks of TAC, respective 3/3/3 mice of each Sham/TAC/raloxifene group were sacrificed after echocardiography, and heart tissues were harvested which were immediately frozen in liquid nitrogen or embedded in paraffin.

### 2.2. Transthoracic Echocardiography Measurement

Respective 3/3/3 mice of each Sham/TAC/raloxifene group at 4 or 8 weeks were performed with echocardiography (Vevo 2100, FUJIFILM VisualSonics, Toronto, Canada) in East Hospital, Tongji University School of Medicine, Shanghai, China. Mice were anesthetized with isoflurane (3% for induction and 2% for maintenance) mixed in 1 L/min 100% O_2_ via a facemask. Cardiac parameters were measured and averaged from at least 3 separate cardiac cycles. The echocardiography operator was blinded to the grouping of mice.

### 2.3. Histology and Immunohistochemistry

The paraffin-embedded tissues were sliced and performed with hematoxylin-eosin (HE), Sirius red, or Masson trichrome staining. The interstitial fields and the perivascular fields containing vasculature were imaged. Immunohistochemistry was performed with antibodies of IL-6 (D220828, Sangon, Shanghai, China), TNF-*α* (bs-2081R, Bioss, Beijing, China), and ANP and MYH7B (ab225844 and ab172967, Abcam, U.S.). The EVOS FL Auto Imaging System (Life Technologies, ThermoFisher Scientific, Waltham, MA, U.S.) was operated to obtain 3-5 random fields of each image.

RETRACTED

### 2.4. Hypertrophic Cell Model and Treatments

H9c2 myoblasts were obtained from the American Type Culture Collection (ATCC, Manassas, U.S.). Cells were cultured in high glucose Dulbecco's modified Eagle's medium (DMEM, KeyGEN BioTECH, Nanjing, Jiangsu, China) supplemented with 10% (*v*/*v*) fetal bovine serum (FBS, Gibco, ThermoFisher Scientific, Waltham, MA, U.S.) and 1% (*v*/*v*) penicillin/streptomycin (Sangon, Shanghai, China) at 37°C in a 5% CO_2_ atmosphere incubator. To induce cellular hypertrophy of H9c2, cells were incubated with IL-6 (No. 200-06, PeproTech, Suzhou, Jiangsu, China, 25 ng/mL), respectively, for 24 h or 48 h, and then, molecular markers were detected by west blotting. To illustrate the effects of raloxifene, H9c2 myoblasts were pretreated with raloxifene (25 *μ*M) for 2 hours and then incubated with IL-6 (25 ng/mL) for 24 h, the cycle was repeated once more (a total of 4 hours for raloxifene and 48 hours for IL-6), and then cells were harvested for staining or western blotting.

### 2.5. Gentian Violet Staining

The cells were treated with IL-6 as above and then were fixed with 4% paraformaldehyde (Sigma-Aldrich) for 20 minutes. The cells were stained with 0.5% (*m*/*v*) gentian violet (ThermoFisher Scientific, Waltham, MA, U.S.) solution for 30 minutes at room temperature and washed twice with PBS. Images were obtained by the EVOS FL Auto Imaging System.

### 2.6. RNA Isolation and Quantitative Real-Time Polymerase Chain Reaction (qRT-PCR)

Total RNA was isolated from frozen heart tissues using the Hipure Total RNA Mini Kit (Magen, Guangzhou, China). The RNA quality and concentration were determined spectrophotometrically (NanoDrop 2000 spectrophotometer, Thermo Scientific, U.S.), and reverse transcription for cDNA synthesis was performed using the ReverTra Ace qPCR RT Kit (TOYOBO Co. Ltd, Osaka, Japan). qPCR was performed with the SYBR green PCR master mix kit (TOYOBO Co. Ltd, Osaka, Japan) on the StepOnePlus real-time PCR system (Applied Biosystems). The mRNA expressions of atrial natriuretic peptide (ANP), B-type natriuretic peptide (BNP), collagen type I alpha 1 (COL1A1), and collagen type III alpha 1 (COL3A1) were normalized to glyceraldehyde-3-phosphate dehydrogenase (GAPDH) by the *ΔΔ*Ct method.

RETRACTED

The primer sequences are listed as follows (mouse): **ANP** forward: 5′-CCT AAG CCC TTG TGG TGT GT, reverse: 5′-CAG AGT GGG AGA GGC AAG AC; **BNP** forward: 5′-CTG AAG GTG CTG TCC CAG AT, reverse: 5′-CCT TGG TCC TTC AAG AGC TG; **COL1A1** forward: 5′-TGA ACG TGG TGT ACA AGG TC, reverse: 5′-CCA TCT TTA CCA GGA GAA CCA T; **COL3A1** forward: 5′-GCA CAG CAG TCC AAC GTA GA, reverse: 5′-TCT CCA AAT GGG ATC TCT GG; **GAPDH** forward: 5′-AGG TCG GTG TGA ACG GAT TTG, reverse: 5′-TGT AGA CCA TGT AGT TGA GGT CA.

### 2.7. Measurement of Intracellular Reactive Oxygen Species (ROS)

The fluorescent dye dihydroethidium (DHE; HY-D0079, MedChemExpress, U.S.) was utilized to evaluate superoxide production in cultured cells. H9c2 myoblasts were treated with IL-6 and raloxifene as described above and then were incubated with 10 *μ*M DHE at 37°C for 30 minutes in the dark and washed twice with PBS. The cells were excited with blue light, and red fluorescence emission images were obtained with the EVOS fluorescence microscope.

### 2.8. Mitochondrial Membrane Potential Measurement

The mitochondrial membrane potential (MMP, *Δ*ᴪ_m_) was monitored by fluorescent probe JC-1 (PJC-110, Promotor Biological Co. LTD., Wuhan, China). H9c2 myoblasts were treated with IL-6 and raloxifene as described above and then were incubated with JC-1 dye for 20 minutes at 37°C and washed twice with PBS. JC-1 was excited at 488 nm, and the red (aggregate) or green (monomer) emission fluorescence was detected with a standard red or green filter by the MShot fluorescence microscope (Wuhan, China).

### 2.9. Measurement of the Total SOD Activity

H9c2 myoblasts were treated with IL-6 and raloxifene as described above and harvested as above. The protein content was measured with the BCA Protein Assay, and then, the activity of total intracellular SOD (superoxide dismutase, units/mg) was analyzed at 450 nm by a microplate reader (TECAN, SUNRISE, Switzerland) using the commercially available kit (Total Superoxide Dismutase Assay Kit, Beyotime, S0101, WST-8) according to the manufacturer's instructions.

### 2.10. The Intracellular Content of ATP Measurement

Intracellular ATP content was measured using a commercially available intracellular ATP Assay Kit (S0026, Beyotime, Shanghai, China) according to the manufacturer's instructions. H9c2 myoblasts were treated with IL-6 and raloxifene as described above and harvested as above. 100 *μ*L ATP detection reagent was added to each well of the 96-well plate and incubated at room temperature for 5 min to minimize the background. 20 *μ*L supernatant was then mixed up with ATP detection reagent in each well, and luminescence (RLU) was measured by a microplate reader (Synergy 2, BioTek Instruments, U.S.). ATP standard curve was used to transform luminescence (RLU) to ATP concentration.

RETRACTED

### 2.11. Protein Extraction and Western Blotting

The pulverized cardiac tissues and the collected cultured cells were lysed in RIPA lysis buffer (Sangon, Shanghai, China) containing 1 mM protease inhibitor and 1 mM phosphatase inhibitor for 40 minutes and centrifuged at 12,000 rpm for 20 minutes at 4°C. The supernatant was collected and quantified by the BCA Protein Assay (Sangon, Shanghai, China). Proteins (25-40 *μ*g) were loaded onto 10% Bis-Tris SDS-polyacrylamide gels and underwent electrophoresis at 60 V for 30 minutes and then 120 V for 1 hour. Then, the separated protein was transferred to 0.45 *μ*m PVDF membranes (Bio-Rad) at 230 mA for 100 minutes. After blocking with TBS-T (Tris-buffer saline containing 0.1% Tween 20) containing 5% powdered milk for 90 minutes, then incubated with primary antibodies overnight, including STAT3 (#4904, Cell Signaling Technology, CST), p-STAT3 (Tyr705) (#9145, CST), p-STAT1 (Tyr701) (#7649, CST), p-STAT5 (Tyr694) (D155020, BBI Life Sciences), PHB2 (#14085, CST), SOD2 (#13141, CST), iNOS (#13120, CST), Pink1 (ab23707, Abcam), Parkin (#4211, CST), Bnip3 (ab10433, Abcam), and GAPDH (10494-1-AP, Proteintech), horseradish peroxidase-conjugated secondary antibodies and Immobilon Western Chemiluminescent HRP Substrate (AntGene Co. Ltd, Wuhan, China) were used for protein detection which was operated on the ChemiDoc-It 510 Imager with VisionWorks software (Ultra-Violet Products Ltd., Cambridge, UK).

### 2.12. Statistical Analysis

SPSS Statistics 25.0 and GraphPad 5.0 were used for statistical analysis and drawing. Continuous variables were expressed as mean ± SEM. Statistical analysis among multiple groups was tested by the one-way analysis of variance (one-way ANOVA) followed with the Bonferroni posttest, and the Mann-Whitney *U* test was used for comparison between two groups. Quantitative assessment of western blotting, immunohistochemistry images, and fluorescence intensity was performed by ImageJ 1.45s. For all statistical analyses, *p* < 0.05 indicates statistical significance.

## 3. Results

### 3.1. Raloxifene Ameliorated Cardiac Hypertrophy Induced by Pressure Overload in TAC Mice

TAC enlarged the murine heart size compared with the Sham group morphologically and histologically, and the heart size was decreased by raloxifene treatment (Figures 1(a) and 1(b)). The cross-sectional area of cardiomyocytes was increased on the transverse-axis view after TAC at both time points, and raloxifene mitigated the hypertrophic response (4 weeks, Sham vs. TAC vs. raloxifene = 1 : 1.32 : 1.02 fold, *p* < 0.01; 8 weeks, Sham vs. TAC vs. raloxifene = 1 : 1.69 : 1 fold, *p* < 0.001) (Figures 1(a) and 1(b)).

RETRACTED

Table 1 shows other parameters that are identified as cardiac hypertrophic indicators in previous studies [17, 20]. Murine heart weight (HW) after TAC at 4 and 8 weeks was significantly increased compared with the Sham group (*p* < 0.05), and raloxifene reduced heart weight compared with the TAC group at both time points (*p* < 0.05). The ratio of HW/body weight (BW) and HW/tibia length (TL) excludes the bias of body weight and was increased in the TAC group compared with that of the Sham group at both time points (*p* < 0.05). But the ratios of the raloxifene group at 8 weeks were both prominently dropped in comparison with the TAC group (*p* < 0.05), whereas the decrease of the HW/BW ratio at 4 weeks showed no difference (*p* = 0.089) (Table 1). Meanwhile, the expression of ANP and MYH7B, which are molecular markers of myocardial hypertrophy [21], in myocardial tissue detected by immunohistochemical staining was increased at both time points, while raloxifene moderated this effect (Figures 1(c) and 1(d)).

### 3.2. Raloxifene Mitigated Pressure Overload-Induced Cardiac Dysfunction in TAC Mice

The left ventricular end-diastolic diameter (LVEDd) and left ventricular end-systolic diameter (LVEDs) of the TAC group at 8 weeks were larger than that of the Sham group or the raloxifene group visually from the images of echocardiography (Figure 2(b)), whereas was not obvious at 4 weeks (Figure 2(a)). The detailed cardiac parameters detected by echocardiography are shown in Table 1. Left ventricular ejection fraction (LVEF) and left ventricular fractional shortening (LVFS) of the TAC group (4 and 8 weeks) were significantly decreased (*p* < 0.05), and raloxifene improved both of them at 8 weeks compared with the TAC group (*p* < 0.05). Other parameters including LVEDd and left ventricular end-diastolic volume (LVEVd), as well as LVEDs and left ventricular end-systolic volume (LVEVs), which reflect systolic function [17], were all significantly increased after TAC operation (8 weeks) compared with the Sham group (*p* < 0.05), but raloxifene ameliorated the deterioration of them compared with the TAC group (*p* < 0.05) (Table 1). However, raloxifene showed no protective effects on cardiac function at 4 weeks because there was no difference between the raloxifene group and the TAC group (Table 1). The ultrasonic parameters, including LVEF, LVEDs, LVEVd, and LVEVs of the 8-week TAC group, also showed that the cardiac function was more severe than that of the 4-week TAC group (Table 1). However, the parameters indicated that the cardiac function of the Sham group or the raloxifene group showed no difference between the two time points (Table 1). The mRNA expressions of BNP and ANP in TAC murine hearts at 8 weeks were abundantly increased compared with the Sham group (ANP, *p* < 0.05; BNP, *p* < 0.001) and were remarkably decreased by raloxifene treatment contrast to the TAC group (ANP, *p* < 0.05; BNP, *p* < 0.001) (Figures 2(c) and 2(d)).

RETRACTED

### 3.3. Raloxifene Prevented Cardiac Fibrosis Induced by Pressure Overload in TAC Mice

Pathological left ventricular remodeling evolved at the late stage of TAC, but cardiac fibrosis has occurred since two weeks after aortic constriction [22]. Cardiac fibrosis detected by Masson staining (left two columns) and Sirius-red staining (right two columns) is shown in Figures 3(a) and 3(b). TAC dramatically exacerbated interstitial and perivascular fibrosis compared with the Sham group at both time points (*p* < 0.05), but raloxifene ameliorated the fibrotic effect of interstitial substance and around the blood vessels at both time points (*p* < 0.05) (Figures 3(c) and 3(d)). Col1A1 and Col3A1 mRNA expressions of murine hearts in the TAC group at 8 weeks were significantly increased compared with the Sham group (*p* < 0.05). Raloxifene downregulated the Col3A1 mRNA expression (*p* < 0.05) while not for Col1A1 (*p* = 0.855) (Figures 3(e) and 3(f)).

### 3.4. Raloxifene Extenuated the Inflammation including Macrophage Infiltration and IL-6 and TNF-*α* Expression in TAC Murine Myocardium

We detected the macrophage marker (CD68) and two crucial cytokines of chronic inflammation (IL-6 and TNF-*α*), in myocardial tissue by immunohistochemical staining. The infiltration of macrophages and the expression of IL-6 and TNF-*α* in murine heart tissues were increased after TAC at both 4 and 8 weeks, which indicated the myocardial inflammation activation by pressure overload. Raloxifene mitigated the increase of CD68, IL-6, and TNF-*α* (Figures 4(a)–4(c)).

### 3.5. Raloxifene Modulated the IL-6/STAT3 Signaling and Inhibited the Phosphorylation of STAT3 in Pressure Overload-Induced Murine Hearts

We detected the protein expression in murine hearts and found that phosphorylation of STAT3 was remarkably increased at both 4 weeks (*p* < 0.001) and 8 weeks (*p* < 0.001) after TAC, and raloxifene decreased the p-STAT3 level significantly at both time points (*p* < 0.01), which indicated the IL-6/STAT3 signaling was activated in TAC murine hearts (Figures 5(a), 5(b), 5(d), and 5(e)). Meanwhile, the expression of PHB2, a mitochondrial structural protein, in the TAC group was increased notably compared with the Sham group (4 weeks, *p* < 0.05; 8 weeks, *p* < 0.01), which was decreased after raloxifene administration (4 weeks, *p* < 0.05; 8 weeks, *p* < 0.001) (Figures 5(c) and 5(f)).

RETRACTED

### 3.6. Raloxifene Inhibited the Activation of IL-6/STAT3 Signaling and Hypertrophic Response Induced by IL-6 in H9c2 Myoblasts

We treated the H9c2 myoblasts with IL-6 (25 ng/mL) continuously for 24 and 48 hours and found that the cell size was enlarged significantly elicited by IL-6 after 48 hours (*p* < 0.001) (Figures 6(a) and 6(b)). The molecular marker of cellular hypertrophy, such as ANP (*p* < 0.05) and MYH7B (*p* < 0.05), was remarkably upregulated after IL-6 incubation for 48 hours (Figures 6(c)–6(e)). Meanwhile, the level of p-STAT3 (48 h, *p* < 0.05) and the expression of PHB2 (48 h, *p* < 0.05) were also concurrently increased in a time-dependent manner (Figures 6(f) and 6(g)), which illustrated that the hypertrophy of H9c2 myoblasts induced by IL-6 accompanied with activation of inflammatory signaling.

Next, we pretreated H9c2 myoblasts with raloxifene (25 *μ*M) and triggered it with IL-6 (25 ng/mL) for 48 hours. The increase of p-STAT3 level and PHB2 expression in H9c2 myoblasts induced by IL-6 was attenuated by raloxifene (p-STAT3, *p* < 0.05; PHB2, *p* < 0.05) (Figures 6(h)–6(j)). This illustrated that the IL-6/STAT3 signaling was inhibited by raloxifene *in vitro*.

### 3.7. Raloxifene Inhibited Oxidative Stress Activation and Regulated Mitophagy-Related Protein Expression Induced by IL-6 in H9c2 Myoblasts

We detected the superoxide production of H9c2 myoblasts by DHE staining and found the fluorescence intensity which indicated the oxidative stress extent of H9c2 cells was increased by sustained IL-6 stimulation (*p* < 0.01) and raloxifene alleviated the effect (*p* < 0.05) (Figures 7(a) and 7(c)). Excessive oxidative stress caused the dysfunction of mitochondria, which might accompany the decrease of mitochondrial membrane potential. JC-1 staining showed that the JC-1 aggregate/monomer ratio decreased after incubation of IL-6 (25 ng/mL) for 48 h and raloxifene reversed the depolarization of MMP (Figures 7(b) and 7(d)). We further detected the ATP content of H9c2 myoblasts and found that the intracellular ATP content was decreased after the continuous incubation of IL-6 for 48 hours compared with the control group, and the ATP content was maintained after pretreating with raloxifene before IL-6 incubation (Figure 7(e)). Meantime, iNOS expression was increased (*p* < 0.001), but the SOD2 expression showed no difference (*p* > 0.99) after IL-6 irritation, but the total intracellular SOD activity was inhibited by IL-6 (*p* < 0.05). Raloxifene significantly increased SOD2 expression (*p* < 0.01), reduced iNOS expression (*p* < 0.001), and increased the SOD activity (*p* < 0.05) (Figures 7(f)–7(h) and 7(l)). These indicated oxidative stress activation by IL-6 was mitigated by raloxifene in H9c2 myoblasts. The excessive oxidative stress activation usually caused the damage of mitochondria and activated mitophagy. The mitophagy-related protein including Pink1 (*p* < 0.05), Parkin (*p* < 0.001), and Bnip3 (*p* < 0.01) was increased after IL-6 stimulation, and raloxifene regulated the protein expression to basic status (Figures 7(i)–7(k)).

RETRACTED

## 4. Discussion

Inflammation underlies a wide variety of physiological and pathological processes [23]. The interaction of inflammation and CVD is the hotspot of the cardiovascular field recently. HF is the end-stage of most CVD, more and more clinical and experimental studies indicate that inflammation takes an important part in the initiation and development of CVD, including atherosclerosis [24], hypertension [25], and atrial fibrillation [26]. Therefore, inflammation might contribute to the initiation, maintenance, and progression of HF. Whereupon, we investigated the role of inflammation in the pressure overload-HF mice and IL-6-elicited H9c2 myoblasts, as well as the anti-inflammatory effect of raloxifene.

In response to the pathogenesis of pressure overload after TAC operation, the heart undergoes cardiac hypertrophy and fibrosis at the late stage, evolving into HF finally, while initially benefitting from compensatory elevation of the cardiac wall tension at the early stage to maintain cardiac function [19, 22]. The heart failure induced by pressure overload through TAC in our study was principally characterized by systolic dysfunction. We compared the difference of tissue features between different stages after TAC. At the early stage (4 weeks), the myocardial hypertrophy and fibrosis have developed but were not conspicuous as compared with that of the late stage (8 weeks). Although the left ventricular dysfunction at 4 weeks was not obvious, inflammation has already been activated at the early stage (4 weeks) and sustained to the late stage (8 weeks), which indicates inflammation might continuously contribute to the HF progression.

Our cooperative group previously found that the N and O of the piperidinyl-ethoxy moiety of raloxifene could form hydrogen bonds with Asn92 and Cys6 residue of gp130 D1 domain, which disrupts the native IL-6 binding interaction with the gp130 [15]. Raloxifene was proved to downregulate the IL-6-induced STAT3 phosphorylation in pancreatic and hepatic cancer cells [15, 16], which indicates that raloxifene is an effective IL-6/gp130 inhibitor. In vitro study, raloxifene was proved to downregulate the STAT3 phosphorylation induced by IL-6 in hepatic cancer cells, but not the induction of STAT1 and STAT6 phosphorylation by IFN-*γ*, IFN-*α*, and IL-4 [16]. Supplementary Figure 1 indicated that raloxifene inhibited the STAT3 phosphorylation induced by IL-6 in H9c2 myoblasts but not by the other cytokines of the IL-6 family, such as LIF and OSM. Meanwhile, the induction of STAT1 and STAT5 phosphorylation induced by IL-6, LIF, and OSM was not inhibited by raloxifene. Hence, we thought that raloxifene was a relatively selective inhibitor of IL-6/gp130/STAT3 signaling. We administrated raloxifene to TAC mice and found that the inflammatory IL-6/gp130/STAT3 signaling was suppressed in murine hearts. Myocardial remodeling was ameliorated at both stages, as well as the cardiac function was partly maintained at the late stage (8 weeks). The animal experiments of our study demonstrated the inflammation was activated in TAC mice, which was consistent with previous research [22, 27]. Previous studies also revealed that the IL-6 level of serum in TAC mice was increased [28] and the IL-10/STAT3 signaling was activated in pressure overload-induced cardiac dysfunction [29]. The previous study reported that IL-6 deletion attenuated the left ventricular hypertrophy and dysfunction induced by 6-week TAC in mice and proved that both angiotensin II- and phenylephrine-induced increase in hypertrophy genes were abrogated in IL-6-/- cardiac myocyte [13]. These indicated that IL-6 is critical to cardiac hypertrophy and dysfunction in response to TAC. However, the genome-editing technique used in human cardiovascular disease therapy is still debatable due to the safety concern and ethical issues; hence, the pharmacological intervention on IL-6/gp130/STAT3 signal by raloxifene is more translatable compared with genome manipulation. Raloxifene might modulate multiple mechanisms, and the IL-6/STAT3 signal might be one of the important options. Our results indicated inhibition of the IL-6/gp130/STAT3 pathway accompanied with the alleviation of the pathological remodeling and heart failure induced by pressure overload; therefore, we thought that the intervention of IL-6/STAT3 signal by raloxifene might involve the pivotal mechanism of the remission. We also found that the local inflammation of heart tissues in TAC mice was increased likewise, IL-6/gp130/STAT3 inhibition related to the mitigation of inflammation and the remission of cardiac remodeling and dysfunction in TAC mice, which was not reported by previous research.

RETRACTED

When the aorta was constricted, fluctuation and overload of blood pressure activated the renin-angiotensin-aldosterone system (RAAS), which initiates a cascade reaction of neurohormone regulation [22]; in this condition, cardiomyocytes and cardiac fibroblasts would release TNF-*α* and IL-6 [22, 30]. The proinflammatory cytokines would orchestrate the expression of cytokines and chemokines and thus promotes the injury of resident interstitial cells and the recruitment of immune cells [22, 31, 32]. The accumulation of abundant inflammatory factors and inflammatory cells provides an inflammatory microenvironment for cardiac remodeling and heart failure. We further found that the phosphorylation of STAT3 in the myocardial tissue of TAC mice was significantly increased and IL-6/gp130/STAT3 inhibition has a cardioprotective effect, all of which indicated that the inflammatory signaling pathway of the IL-6/gp130/STAT3 axis might play a crucial role in the cardiac remodeling and HF. Moreover, inflammation promoted excessive ROS production, which was proved to damage the mitochondrial homeostasis and cause energy metabolism disorder [33].

High energy demand, especially the high ATP consumption, is one of the major features of the heart, and oxidative metabolism in the mitochondria is the predominant derivation of ATP production [34]. The oxidative phosphorylation takes place in the inner mitochondrial membrane; hence, the inner membrane integrity and the mitochondrial membrane potential are critical for mitochondrial function [34]. PHB2 is involved in the electron transport chain and maintains the structure and function of mitochondria [35], and it could translocate to the nucleus and participate in oxidative stress and apoptosis [36]. Theiss et al. reported that STAT3 mediated IL-6-induced PHB transcription and bound to the IL-6 response element in its promoter [37], but the concrete role of PHB2 in myocardial hypertrophy is unsettled [38, 39]. In our study, the PHB2 expression was increased in TAC-induced murine heart and IL-6-elicited H9c2 myoblasts and was decreased by raloxifene treatment. Importantly, the alteration of PHB2 was consistent with the phosphorylation of STAT3. Meantime, the superoxide productions triggered by IL-6 in H9c2 myoblasts were inhibited by raloxifene, the depression of mitochondrial membrane potential induced by IL-6 was reversed by raloxifene, and the ATP content was maintained after pretreating with raloxifene before IL-6 incubation. IL-6 induced the oxidative stress producer (iNOS) increase and scavenger (SOD2) decrease in H9c2 myoblasts, which was reversed by raloxifene. These results indicated that raloxifene could exert the cardioprotective effect via mitigating oxidative stress-induced mitochondrial dysfunction on H9c2 myoblasts induced by continuous IL-6 incubation.

As reported, the damaged mitochondria would release cytochrome C and thereby trigger apoptosis. The appropriate elimination of dysfunctional mitochondria is essential to cellular survival [40]. Mitophagy is an important control mechanism for regulating the adjustments to mitochondrial status with oxidative stress [41], and mitophagy is found to play a protective role in most cardiovascular disease [42]. As our results were shown, two classic mediators of mitophagy, Pink1 and Parkin, were increased by sustained IL-6 incubation. The disturbance of MMP leads to PINK1 accumulation at the surface of the mitochondria, promoting the subsequent recruitment of Parkin, which is the initiation of the classic Pink/Parkin-dependent pathway in mitophagy [43]. Meanwhile, the expression of Bnip3, which plays a critical role in the mitophagy receptor-dependent pathway, was also increased after IL-6 stimulation. Excessive activation of autophagy elicited by pathological stimuli, such as pressure overload, is maladaptive and promotes cell apoptosis, which was reported to aggravate cardiac hypertrophy and speed up the process of HF [44]. Mitophagy, as a selective autophagy, is activated in the early stage of cardiac hypertrophy during HF, which ultimately promotes cell apoptosis [45]. Hence, the proper mitophagy is imperative for cellular survival. We found that raloxifene decreased the expression of Pink1, Parkin, and Bnip3 elicited by IL-6 stimuli, which indicated that the biological effect of raloxifene was involved in the mitochondrial quality control by resuming the increase of mitophagy-related proteins induced by excessive ROS and the loss of MMP. Hence, TAC-induced hemodynamic changes activate inflammation especially the IL-6/STAT3 signaling, as well as the production of reactive oxygen species and subsequent imbalance of mitochondrial homeostasis. In turn, excessive ROS could aggravate the inflammation and HF progress as reported [46, 47], which constitutes to a vicious circle of proinflammatory microenvironment. Raloxifene could block the overactivated IL-6/STAT3 signaling and alleviate the inflammation with decreased oxidative stress and regulation of the mitophagy level.

RETRACTED

Previous studies reported the debatable effect of raloxifene. Ogita et al. found that raloxifene prevented cardiac hypertrophy and dysfunction in pressure overload male mice (4 weeks) [18]. However, Westphal et al. reported that raloxifene was not able to reduce the myocardial remodeling and could not maintain EF in female TAC mice at the long-term period (9 weeks) [17]. The severity of cardiac remodeling and heart failure of the TAC model was influenced by multiple factors and depended on the murine strain, sex, and needle size used for TAC operation [20]. The basal line of cardiac function of mice in different studies might be variant, but the main difference between the two studies was the size of a gauge needle used for TAC operation. Ogita et al. adopted the 27-gauge needle, while Westphal et al. used the 26-gauge needle (the outside diameter was larger than that of the 27-gauge needle) for operation. The previous study by Richards et al. explored the influence of gauge (G) of needle used on the TAC severity [21] and found that the 27G TAC group had more severe systolic and diastolic dysfunction, severe cardiac fibrosis, and was more likely to display features of heart failure compared with the 26G TAC group [21]. Therefore, the severity of phenotype was more obvious in the study of Ogita et al., and the cardioprotective effect of raloxifene might be easier to be observed. Intriguingly, although the pathological cardiac remodeling process might progress at different rates or degrees, the cardiac response to various degrees of pressure overload might not be graded or step-wise [21]. Richards et al. observed that several parameters such as fractional shortening, ejection fraction, and perivascular fibrosis were mixed responses, rather than step-wise [21]. The complexity of TAC operation produced unique pathological phenotypes in different studies. In our study, we used the 27^1/2^-gauge needle (the outside diameter was smaller than that of the 27-gauge needle) for TAC operation; hence, the pathological remodeling and cardiac dysfunction might be more significant than the previous studies, and we also found that raloxifene decelerated the deterioration of heart dysfunction and mitigated the cardiac remodeling and myocardial inflammation in mice induced by TAC to a certain degree at both four and eight weeks. Moreover, the mechanism of the previous study about the effects of raloxifene on TAC mice focused on the activity of MAPK signaling [18] but paid less attention to the motivation of inflammation. In this study, we not only provide more evidence about the cardioprotective effect of raloxifene on TAC mice and we newly found that inflammation and IL-6/gp130/STAT3 signaling were activated in TAC murine heart but inhibited by raloxifene accompanied by the improvement of cardiac hypertrophy and heart failure, which is the mechanism of raloxifene differing from that of the others. On the other hand, the possible reason for the divergence in the previous findings is that there was gender difference in the mouse model of pathological hypertrophy and HF, in which male mice showed more eccentric hypertrophy and HF signs than female mice [48]. Meanwhile, the gender difference in the treatment of raloxifene to rat pulmonary arteries and veins was reported by a previous study [49]. The other study also reported that the production of proinflammatory cytokines, such as IL-6, IL-1*β*, and TNF-*α*, was more obvious in male mice than that in female mice after lipopolysaccharide (LPS) induction [50]. All evidence above indicated that gender might be involved in the effect of TAC or raloxifene, and the inflammatory response of mice. Hence, male mice might be more sensitive to TAC surgery and show serious inflammation, so the effect of raloxifene on male mice might be more significant. These reported results all suggested that inflammation might play a very important role in the progression of cardiac remodeling and HF. Our data not only showed more evidences but also illustrated that the potential inflammatory pathways might include IL-6/gp130/STAT3 signaling.

RETRACTED

Other small molecule STAT3 inhibitor S31-201 [51] was also documented to reduce phosphorylation of STAT3 in Wistar rats induced by renal artery ligation. Meanwhile, the natural product, such as stachydrine [52], celastrol [53], and gallic acid [54], ameliorated isoproterenol- or TAC-induced cardiac hypertrophy, fibrosis, and cardiac dysfunction by inhibiting STAT3 signaling pathways, but the authors did not explore the underlying mechanism. We used raloxifene as an IL-6/STAT3 inhibitor to evaluate its cardioprotective effect on TAC-induced cardiac hypertrophy, heart failure, and myocardial inflammation. Unlike the previous studies, we not only focused on exploring the IL-6/STAT3 signaling pathway but also further evaluated the regulation of raloxifene on the oxidative stress and mitophagy levels induced by continuous inflammatory activation. Raloxifene is also approved by the FDA, and the safety for humans is validated and accepted. The limitation of this research lies in that we did not investigate the further mechanism of how IL-6 regulates mitochondrial homeostasis in the context of TAC-induced HF. To date, the role of IL-6 in the CVD during the acute and chronic phases has been debatable, so the role of IL-6 in the acute phase to heart failure induced by pressure overload is unsettled. Therefore, further studies focused on mitochondrial energy metabolism, mitochondrial quality control, and the relationship between IL-6 were needed to illustrate the detailed mechanism.

## 5. Conclusions

Overall, during the chronic stage of pressure overload-induced heart failure, the expression of IL-6 was upregulated, which activated gp130/STAT3 signaling and produced excessive ROS. Oxidative stress aggravated depolarization of MMP and the damage of mitochondria, which affected the homeostasis of mitochondrial structure and increased the expression of the mitophagy-related proteins, thus resulting in more ROS production and uncontrolled inflammation. The vicious circle could be suppressed via IL-6/gp130 inhibitor, raloxifene, by prohibiting the binding between IL-6 and gp130, which indicated that the IL-6/gp130/STAT3 axis might be involved in the pathogenesis of myocardial hypertrophy and HF.

RETRACTED

## Figures and Tables

**Figure 1:** Raloxifene mitigated murine cardiac hypertrophy induced by TAC. (a, b) Gross morphology of murine heart, transverse sections, and typical regional enlarged images showed cardiac hypertrophy induced by TAC through HE staining. The respective histogram showed the cross-section area of cardiomyocytes enlarged and raloxifene alleviated the hypertrophic response. (c, d) The increased ANP (c) and MYH7B (d) expression of myocardial tissues after TAC of 4 or 8 weeks detected by immunohistochemistry was mitigated by raloxifene. The minimal interval of scale in the three rows of (a) and (b) is 1 mm, 0.5 mm, and 100 *μ*m, respectively, and 100 *μ*m of (c) and (d). ^∗^*p* < 0.05; ^∗∗^*p* < 0.01; ^∗∗∗^*p* < 0.001.

**Figure 2:** Raloxifene reversed the cardiac dysfunction of pressure overload mice. (a, b) M-mode echocardiography images of mice measured at 4 (a) or 8 (b) weeks after TAC. (c, d) The increased mRNA expression of ANP (c) and BNP (d) in the murine hearts at 8 weeks were both reduced by raloxifene treatment. ^∗^*p* < 0.05; ^∗∗∗^*p* < 0.001.

**Figure 3:** Raloxifene alleviated cardiac fibrosis induced by pressure overload. (a, b) The interstitial and perivascular fibrosis of murine hearts increased by Masson staining (left two columns) and Sirius red staining (right two columns) after TAC of 4 (a) or 8 (b) weeks and was alleviated by raloxifene (scale bar, 200 *μ*m). (c, d) The respective histogram exhibited the quantitation for the cardiac fibrosis area of murine hearts at 4 (c) or 8 (d) weeks after TAC. (e, f) Relative Col1A1 (e) and Col3A1 (f) mRNA expression normalized to GAPDH increased in murine hearts after TAC of 8 weeks and was reduced by raloxifene. ^∗^*p* < 0.05; ^∗∗^*p* < 0.01; ^∗∗∗^*p* < 0.001, “ns” stands for “none significance”.

**Figure 4:** Raloxifene alleviated the increase of inflammatory markers in murine myocardial tissues induced by TAC. The local CD68 (a), IL-6 (b), and TNF-*α* (c) expression of myocardial tissues detected by immunohistochemistry after TAC operation and raloxifene treatment of 4 and 8 weeks (scale bar, 200 *μ*m for 20x, 100 *μ*m for 40x). ^∗^*p* < 0.05; ^∗∗^*p* < 0.01; ^∗∗∗^*p* < 0.001.

**Figure 5:** Raloxifene decreased the phosphorylation of STAT3 and the expression of PHB2 in TAC murine heart. The p-STAT3 level, and protein expression of STAT3, PHB2 in murine hearts at 4 (a) and 8 (d) weeks by western blotting, and relative quantitation of p-STAT3 (b, e) and PHB2 (c, f) normalized by GAPDH (*n* = 3 per group). ^∗^*p* < 0.05; ^∗∗^*p* < 0.01; ^∗∗∗^*p* < 0.001.

RETRACTED

**Figure 6:** Raloxifene repressed the phosphorylation of STAT3 in hypertrophic H9c2 myoblasts. (a, b) The gentian violet staining showed H9c2 myoblasts manifested hypertrophy (a) and the relative cell area was increased (b) after incubation with IL-6 (25 ng/mL) for 48 h. (c–g) The sustained IL-6 incubation increased the protein expression of MYH7B (d), ANP (e), PHB2 (f), and the p-STAT3 level (g) in H9c2 myoblasts analyzed by western blotting (c). (h–j) Raloxifene decreased the level of p-STAT3 (i), and the expression of PHB2 (j) in H9c2 myoblasts induced by IL-6. ^∗^*p* < 0.05; ^∗∗^*p* < 0.01; ^∗∗∗^*p* < 0.001, “ns” stands for “none significance”.

**Figure 7:** Raloxifene reduced oxidative stress and regulated mitophagy-related protein expression elicited by IL-6 in H9c2 myoblasts. (a, c) The DHE staining (a) showed that raloxifene alleviated reactive oxygen species production induced by IL-6 (scale bar: 1000 *μ*m for 4x; 200 *μ*m for 20x) and the bar graph (c) showing the mean DHE fluorescence intensity of nuclei in H9c2 myoblasts. (b, d) The JC-1 staining (b) showed that raloxifene reversed the decrease of mitochondrial membrane potential elicited by IL-6 (scale bar, 400 *μ*m); red fluorescent (aggregate)/green fluorescent (monomer) ratio (D) was decreased with the IL-6 incubation and was reversed by raloxifene treatment. (e) The intracellular ATP content was decreased after the continuous incubation of IL-6 for 48 hours but was maintained after pretreating with raloxifene before IL-6 incubation. (f–k) Raloxifene increased the antioxidative protein SOD2 expression (h) and decreased the prooxidative protein iNOS expression (g) of H9c2 myoblasts incubated with IL-6. Meanwhile, raloxifene regulated the mitophagy-related protein of Pink1 (i), Parkin (j), and Bnip3 (k) to normal status. (l) The sustained IL-6 stimulation decreased the total intracellular SOD protein activity and was reversed by raloxifene treatment. ^∗^*p* < 0.05; ^∗∗^*p* < 0.01; ^∗∗∗^*p* < 0.001, “ns” stands for “none significance”.

**Table 1:** LV hypertrophy and dysfunction in murine hearts of four and eight weeks after TAC.

	4 weeks			8 weeks		
	Sham	TAC	TAC+raloxifene	Sham	TAC	TAC+raloxifene
*N*	3	3	3	3	3	3
HW (mg)	101.59 ± 1.24	176.93 ± 5.82^∗^	124.27 ± 6.20^†^	136.83 ± 4.99	237.13 ± 14.66^#,@^	147.30 ± 6.51^$^
HW/BW (mg/g)	4.17 ± 0.06	7.28 ± 0.46^∗^	5.62 ± 0.39	5.03 ± 0.16	8.66 ± 0.51^#^	5.63 ± 0.56^$^
HW/TL (mg/mm)	4.57 ± 0.02	7.80 ± 0.11^∗^	5.49 ± 0.28^†^	6.42 ± 0.24	11.08 ± 0.37^#,@^	6.85 ± 0.54^$^
LVEF (%)	78.36 ± 2.18	63.07 ± 2.52^∗^	61.50 ± 3.41	77.14 ± 3.20	37.09 ± 2.80^#,@^	68.91 ± 6.58^$^
LVFS (%)	45.65 ± 2.23	33.55 ± 1.84^∗^	32.20 ± 2.31	44.89 ± 2.87	16.90 ± 1.77^#^	38.79 ± 5.58^$^
LVEDd (mm)	3.21 ± 0.13	3.67 ± 0.16	3.42 ± 0.08	3.19 ± 0.04	4.39 ± 0.03^#^	3.45 ± 0.18^$^
LVEDs (mm)	1.79 ± 0.13	2.44 ± 0.12	2.30 ± 0.14	1.76 ± 0.11	3.64 ± 0.08^#,@^	2.14 ± 0.29^$^
LVEVd (*μ*L)	41.72 ± 4.04	57.45 ± 5.97	44.12 ± 5.83	40.72 ± 1.34	87.04 ± 1.26^#,@^	49.70 ± 6.02^$^
LVEVs (*μ*L)	14.13 ± 1.18	21.16 ± 2.51	17.53 ± 3.43	12.17 ± 1.17	56.20 ± 3.02^#,@^	16.62 ± 4.85^$^

HW = heart weight; BW = body weight; TL = tibia length; LVEF = left ventricular ejection fraction; LVFS = left ventricular fractional shortening; LVEDd/LVEDs = left ventricular end-diastolic/systolic diameter; LVEVd/LVEVs = left ventricular end-diastolic/systolic volume; ^∗^4 weeks: TAC group vs. Sham group, *p* < 0.05; ^†^4 weeks: TAC+raloxifene group vs. TAC group, *p* < 0.05; ^#^ 8 weeks: TAC group vs. Sham group, *p* < 0.05; ^$^8 weeks: TAC+raloxifene group vs. TAC group, *p* < 0.05; ^@^4 weeks vs. 8 weeks of the indicated group (Sham, TAC, or TAC+raloxifene group), *p* < 0.05.

RETRACTED

## Data Availability

All datasets generated for this study are included in the article.

## Supplementary Materials

Supplementary Materials Supplemental Figure 1: raloxifene relative selectively inhibited the phosphorylation of STAT3 induced by IL-6. Raloxifene (25 *μ*m, 4 h) inhibited the STAT3 phosphorylation induced by IL-6 (25 ng/mL, 30 min) in H9c2 myoblasts, but not STAT1 and STAT5 phosphorylation. The phosphorylation of STAT1, STAT3, and STAT5 induced by the other cytokines of the IL-6 family, such as LIF (25 ng/mL, 30 min) and OSM (25 ng/mL, 30 min), was not inhibited by raloxifene.
